# TP53 regulates human AlkB homologue 2 expression in glioma resistance to Photofrin-mediated photodynamic therapy

**DOI:** 10.1038/sj.bjc.6605797

**Published:** 2010-07-27

**Authors:** S Y Lee, S K Luk, C P Chuang, S P Yip, S S T To, Y M B Yung

**Affiliations:** 1 Department of Health Technology and Informatics, The Hong Kong Polytechnic University, Hung Hom, Kowloon, Hong Kong Special Administrative Region, China

**Keywords:** TP53, ALKBH2, DNA repair, Photofrin, photodynamic therapy

## Abstract

**Background:**

Photodynamic therapy (PDT) is a promising adjuvant therapy in cancer treatment. However, cancers resistant to PDT, mediated through the efflux of photosensitisers by means of P-glycoprotein or ATP-binding cassette transporter proteins, have been reported. The DNA repair has also been suggested to be responsible for PDT resistance, but little is known about the repair pathways and mechanisms involved. Therefore, this study aimed to investigate the possible function of six major DNA repair mechanisms in glioma cells resistant to Photofrin-mediated PDT (Ph-PDT).

**Methods:**

The U87 glioma cells relatively resistant to Ph-PDT were obtained by recovering the viable cells 3 h after PDT treatment. The mRNA and protein expression levels of DNA repair genes were evaluated by quantitative real-time reverse transcription-polymerase chain reaction and western blotting, respectively. Small-interfering RNA and chromatin-immunoprecipitation assays were used to further examine the relationship between AlkB, an alkylation repair homologue 2 (*Escherichia coli*) (*ALKBH2*) and Ph-PDT responsiveness, and transcription factors involved in *ALKBH2* transcription.

**Results:**

The *ALKBH2* of DNA damage reversal was significantly increased at both mRNA and protein levels from 30 min to 48 h post-treatment with Ph-PDT. Conversely, down-regulating *ALKBH2* expression enhances Ph-PDT efficiency. Furthermore, our data clearly show for the first time that tumour protein (TP53) is directly involved by binding to the promoter of *ALKBH2* in mediating Ph-PDT resistance.

**Conclusion:**

C The DNA damage reversal mechanisms may have important functions in Ph-PDT resistance through the activation of *ALKBH2* by TP53.

Glioblastoma multiforme is one of the most common tumours affecting the brain and notoriously difficult to cure. It is because glioma cells are particularly resistant to therapy and coupled with the problem of the blood–brain barrier, and the susceptibility of healthy brain tissue to damage during treatment, new adjuvant therapies are clearly needed to tackle this treatment-resistant tumour (Gerstner and Fine, 2007).

Photodynamic therapy (PDT) is an emerging adjuvant therapy used in the treatment of different tumours (O’Connor *et al*, 2009). The PDT has several advantages over traditional treatment regimens. Compared with surgery and radiotherapy, PDT causes less severe long-term morbidity with comparable treatment outcomes (Nyst *et al*, 2009). It can also be the choice of re-treatment in cases of recurrence and incomplete tumour responses after standard therapies and/or PDT as PDT does not compromise re-treatment effectiveness (Hornung *et al*, 1998).

The PDT uses the excitation of photosensitisers in tumour cells by light to interact with the oxygen in tissues, thus reactive oxygen species are produced to kill the tumour cells through apoptosis or necrosis (Pervaiz, 2001). Photofrin is the most commonly used photosensitiser, and Photofrin-mediated PDT (Ph-PDT) has already been approved for the treatment of different solid tumours by the US Food and Drug Administration (Biel, 2006). Clinical trials using Photofrin to treat gliomas are being carried out, but reports on glioma cell resistance to Ph-PDT *in vitro* or *in vivo* are emerging (Adams *et al*, 1999; Ferrario *et al*, 2007). This situation is also seen in head and neck dysplasia or cancer patients in which some of them failed to respond, or only partially responded to Ph-PDT (Stylli *et al*, 2004; Rigual *et al*, 2009). The underlying cellular mechanisms leading to failure to respond to Ph-PDT are not fully understood. Several proteins and signalling pathways, such as activation of anti-apoptotic proteins, cellular antioxidant defence mechanisms and efflux of photosensitisers by means of P-glycoprotein or ATP-binding cassette transporter proteins have been shown to have significant functions in cellular resistance to Ph-PDT (Saczko *et al*, 2007a; Usuda *et al*, 2008, 2010; Zheng *et al*, 2008). The interactions of these different pathways and proteins may enhance tumour cell proliferation and differentiation, promote invasion and prevent apoptosis, leading to the decreased cytotoxicity of Ph-PDT.

The DNA repair has been shown to reduce cell death caused by different cancer therapies, including radiotherapy and chemotherapy using a platinum agent (Frosina, 2009; Fukushima *et al*, 2009). The Ph-PDT has also been reported to induce significant DNA damage and repair in different cell types (Woods *et al*, 2004; Saczko *et al*, 2008). Although different mechanisms have been suggested to explain the causes of resistance in Ph-PDT, the function of DNA repair mechanisms has not been fully investigated. Therefore, we carried out a series of experiments to investigate the DNA repair mechanism(s) that may be responsible for the survival of glioma cells after Ph-PDT. Specific genes representative of the main DNA repair pathways in human beings were examined. The six specific genes are (1) AlkB, alkylation repair homologue 2 (*Escherichia coli*) (*ALKBH2*) of direct DNA damage reversal; (2) APEX nuclease (multifunctional DNA repair enzyme) 1 (*APEX1*) of base excision repair (BER), which removes small base lesions; (3) X-ray repair complementing defective repair in Chinese hamster cells 1 (*XRCC1*) of short-patch BER, which is responsible for repairing single base damage; (4) excision repair cross-complementing rodent repair deficiency, complementation group 5 (*ERCC5*) of nucleotide excision repair (NER) that repairs bulky, helix-distorting lesions NER; (5) RAD52 homologue (*Saccharomyces cerevisiae*) (*RAD52*) of double-strand break repair and (6) REV1 homologue (*S. cerevisiae*) (*REV1*) of translesion synthesis, which is a DNA damage tolerance machinery (Christmann *et al*, 2003).

In this study, viable glioma cells recovered 3 h after Ph-PDT were considered as relatively resistant/less responsive to Ph-PDT. The gene *ALKBH2*, involved in DNA damage reversal, was significantly expressed in these cells for at least 24 h after Ph-PDT. Knockdown of *ALKBH2* intensified the cytotoxic effect of Photofrin, which implies that it confers resistance to Ph-PDT. We also showed both mRNA and protein levels of *ALKBH2* were up-regulated. This up-regulation was due to the binding of the transcription factor tumour protein (TP53) to one of the predicted promoter regions of *ALKBH2*, a finding that has not been reported before.

## Materials and methods

### Cell culture

The human glioblastoma U87 cell line was obtained from American Type Culture Collection (Rockville, MD, USA). The cells were maintained in Minimum Essential Medium Alpha (Invitrogen, Carlsbad, CA, USA) supplemented with 10% foetal bovine serum (complete medium) and were grown in a humidified atmosphere at 37°C and 5% CO_2_.

### Photosensitiser and photodynamic treatment

Photofrin was a generous gift from Axcan Pharma (Quebec, Canada). Stock solution (2.5 mg ml^−1^) was prepared in 5% dextrose and kept at −20°C until use. Cells (2 × 10^5^) were seeded onto 60 mm culture dishes in complete medium and incubated overnight. Cells were then incubated in serum-free medium containing 1 *μ*g ml^−1^ Photofrin for at least 18 h to achieve maximal uptake before being illuminated (Ph-PDT) (Jiang *et al*, 2003; Dysart and Patterson, 2005; Au *et al*, 2006). Light irradiation of cells was carried out using a quartz-halogen lamp coupled with a 500 nm long-pass filter. The energy fluence rate was 33.5 mW cm^−2^ at a wavelength of 630 nm. The following controls were also included in all experiments: cell cultures without Photofrin and light irradiation (no treatment controls); without Photofrin, but illuminated (light controls, LCs) and with Photofrin, but not illuminated (dark controls, DCs). Three hours after light irradiation, the cells were used directly for cell survival and alkaline comet assays (for examining DNA damage) or allowed to recover in complete medium for various times before being analysed by (i) chromatin immunoprecipitation (ChIP), (ii) western blotting, (iii) real-time quantitative reverse transcription-polymerase chain reaction (RT–PCR) and (iv) alkaline comet assay (for examining DNA repair).

### Cell survival assay

Cell survival was determined using the trypan-blue exclusion method. Cells were diluted 1 : 9 in 500 *μ*l phosphate-buffered saline (PBS) and stained with trypan blue. They were then analysed using an automated Vi-CELL cell viability analyser (Beckman Coulter, Brea, CA, USA), which has linearity approximately from 5 × 10^4^ to >1 × 10^7^ cells ml^−1^ (Szabo *et al*, 2004). The number of viable cells in 50 images was counted and three replicates were performed on each sample.

### Alkaline comet assay

The assay was performed according to an earlier described procedure (Collins *et al*, 1997). In brief, 4 × 10^4^ cells were mixed with 60 *μ*l of 1% low melting point agarose in PBS (37°C) and embedded on an agarose pre-treated standard microscope slide. The slides were then immersed in lysis buffer for 1 h to denature the cellular proteins and then transferred to the alkaline electrophoresis buffer and incubated for 30 min at 4°C in the dark for DNA unwinding. Electrophoresis was then conducted for 30 min at 25 V and 300 mA. Slides were neutralised with three changes of 0.4 M Tris–HCl buffer, pH 7.5, for 5 min each and stained with 30 *μ*l ethidium bromide (20 *μ*g ml^−1^). Individual comets were viewed at a final magnification of × 400 using a fluorescence microscope (Eclipse E600, Nikon, Tokyo, Japan) equipped with 590 nm long-pass emission filter. Comets from two slides of each sample were analysed using the Komet 5.5 software (Kinetic imaging, Liverpool, UK) and 150 individual comets were counted.

### Real-time quantitative RT–PCR

Total RNA was isolated using PureLink Micro-to-Midi Total RNA Purification kit (Invitrogen), and reverse transcribed using RevertAid First Strand cDNA Synthesis kit (Fermentas, Ontario, Canada) with oligo-dT primers according to the manufacturers’ protocols. To analyse the relative gene expression, cDNA was then subjected to TaqMan-based real-time quantitative PCR in a 7500 Real-Time PCR system (Applied Biosystems, Foster City, CA, USA). Briefly, 7.5 ng of cDNA were added to 20 *μ*l of PCR mix containing 1 × Universal PCR Master Mix and 1 *μ*l validated TaqMan gene expression assay mix (Applied Biosystems) for each gene shown in Table 1. The amplification was carried out as follows: 1 cycle for denaturation (95°C per 10 min) followed by 40 cycles for two-stage PCR (95°C per 15 s and 60°C per 1 min). Fluorescence signals were measured continuously during the repetitive cycles. The relative changes in gene expression were calculated based on the 2^−ΔΔCt^ method (Livak and Schmittgen, 2001).

### Western blotting

Cells were collected, washed in ice-cold PBS and lysed in WCE buffer (20 mM HEPES, 1 mM EDTA, 1 mM EGTA, 0.2 M NaCl, 0.5% Triton X-100, 10% glycerol and complete mini protease inhibitor cocktail tablet (Roche, Branchburg, NJ, USA)). The lysates were boiled in SDS sample buffer (62.5 mM Tris–HCl (pH 6.8), 1% *β*-mercaptoethanol, 10% glycerol, 1% SDS and 0.001% bromophenol blue) and separated by 10% SDS–PAGE. The separated proteins were then blotted onto PVDF membranes (Amersham Biosciences, Uppsala, Sweden) and blocked with 5% non-fat milk or 5% bovine serum albumin (for Phospho-p53 antibody) in Tris-buffered saline (pH 7.4) containing 0.1% Tween 20 for 1 h at room temperature. To examine different protein expression, the membranes were probed with antibodies against ALKBH2 (1 : 1000 dilution, Abcam, Cambridge, UK), REV1 (1 : 500 dilution, Abcam), NPM/B23 (1 : 1000 dilution), p53 (1 : 200 dilution, Santa Cruz Biotechnology, Santa Cruz, CA, USA), Phospho-p53 (Ser-15) (1 : 1000 dilution, Cell Signaling Technology, Beverly, MA, USA) and *β*-actin (1 : 2000 dilution, Santa Cruz Biotechnology). Corresponding horseradish peroxidase-labelled anti-rabbit and anti-mouse antibodies were used as secondary antibodies (Cell Signaling Technology). The final complexes were visualised by enhanced chemiluminescence autoradiography (Perkin Elmer, Cambridge, MA, USA).

### Small-interfering RNA transfection

Fifty per cent confluent density of U87 glioma cells (1 × 10^5^) were seeded onto 35 mm dishes in complete medium and incubated overnight. Small-interfering RNA (siRNA) oligomers and Lipofectamine 2000 transfection reagent (100 pmol and 1 : 50 dilution, respectively, Invitrogen) were mixed with serum-free medium, incubated and added to each dish. In mock controls, the negative control RNA was used instead of siRNA to act as a control. Cells incubated with Lipofectamine alone were used as reagent control. After 6 h of incubation, the cells were recovered in complete medium for 16 h. They were then subjected to Ph-PDT treatment as described above. Three hours after light irradiation, cells were analysed by real-time quantitative RT–PCR, western blotting and cell survival assay.

### Chromatin immunoprecipitation

The U87 glioma cells were allowed to recover for 6 h after Ph-PDT. They were then cross-linked by formaldehyde (1% final concentration) at room temperature for 10 min. The fixation was quenched by the addition of glycine at a final concentration of 0.125 M. The cells were washed with cold PBS containing protease inhibitors (Roche) and collected by scraping. The ChIP was performed using the MAGnify chromatin-immunoprecipitation system (Invitrogen) according to the manufacturer's protocol. Briefly, the cells were lysed and chromatin was released from the nuclei. Chromatin was sheared to around 200 to 500 bp fragment sizes by sonication. The cross-linked protein–protein and protein–DNA fragments were immunoprecipitated by anti-TP53 or anti-IgG antibodies conjugated to Dynabeads Protein A/G. The cross-linking was reversed by heat treatment, and DNA associated with TP53 was isolated by DNA purification magnetic beads. The isolated DNA was analysed by both conventional and real-time PCR.

### PCR analysis for ChIP

The primers (Table 2) for conventional and SYBR green real-time quantitative PCR were designed from *Homo sapiens* chromosome 12 reference complement sequence (accession no: NC_000012.10) using the Oligo program version 6.57 (Molecular Biology Insights, Cascade, CO, USA). In conventional PCR, 5 *μ*l of each DNA sample from ChIP assay were mixed with 25 *μ*l of PCR master mix containing 1X GeneAmp PCR Gold Buffer, 0.2 mM of each dNTP, 2.5 mM MgCl_2_, 0.3 *μ*M of each primer and 0.5U AmpliTaq Gold DNA polymerase (Applied Biosystems). The amplification cycle was carried out as follows: 1 cycle for denaturation (95°C per 5 min) followed by 30 cycles for amplification (95°C per 15 s, 55°C per 1 min and 72°C per 1 min) and final extension of 10 min at 72°C. The PCR products were subjected to agarose gel electrophoresis for examination. In real-time quantitative PCR using SYBR green, 5 *μ*l of each DNA sample were mixed with 25 *μ*l of PCR mix containing Maxima SYBR Green/ROX qPCR Master Mix (Fermentas) and 0.3 *μ*M of each primer. The amplification cycle used was as follows: 1 cycle for denaturation (95°C per 10 min) followed by 40 cycles for amplification (95°C per 15 s and 60°C per 1 min). Fluorescence signals were measured continuously during the repetitive cycles with an Applied Biosystems 7500 Real-Time PCR system. The relative changes in gene expression were calculated based on the 2^−ΔΔCt^ method.

### Statistics

Data are presented as mean+s.d. Statistical significance for differences was determined by paired *t*-test, one-way ANOVA with Tukey's post-test and two-way ANOVA with Bonferroni's post-test.

## Results

### Photofrin-mediated photodynamic treatment causes DNA damage

The U87 glioma cells without Photofrin treatment were exposed to different light doses, namely control (CNT) at 0 J cm^−2^, LC 1 at 0.8 J cm^−2^ and LC 2 at 1.3 J cm^−2^, respectively. The mean DNA percentage in comet tails of LCs (∼2%) was not significantly different from CNT (Figure 1). When cells were treated with Photofrin (1 *μ*g ml^−1^) and exposed to different light doses (DC at 0 J cm^−2^, lethal dose (LD) 10 at 0.8 J cm^−2^ and LD 40 at 1.3 J cm^−2^), there was significant DNA damage as the mean DNA percentage in comet tails increased 3 h (black bars in Figure 1) after light irradiation (8.1% in DC, 13.9% in LD 10 and 33.2% in LD 40; all *P*<0.001 when compared with that of CNT). Photofrin alone caused DNA damage and light activation caused further DNA damage in a light dose-dependent manner.

### Involvement of DNA repair in relatively resistant glioma cells after recovery from Ph-PDT

To determine whether there was any DNA repair in the relatively resistant glioma cells that survived Ph-PDT, DNA damage was evaluated after the cells had been allowed to recover for 24 h. There was no significant change in the mean DNA percentage in comet tails of CNT and LCs. In contrast, the mean DNA percentage of DC (3.3%), LD 10 (10.3%) and LD 40 (20.3%) were reduced considerably when compared with those cells that had recovered for 3 h only (white bars compared with black bars in Figure 1).

### *ALKBH2* expression increases significantly after recovery from Ph-PDT

The involvement of the six selected DNA repair pathways were evaluated by determining the relative mRNA expression levels (−ΔΔCt) of their target DNA repair genes in the less responsive glioma cells, that is surviving cells after Ph-PDT, 48 h after treatment. Most of the target genes were expressed equally in both control and treated cells (Figure 2A). However, *ALKBH2* and *REV1* were significantly over-expressed in those LD 10 and LD 40 recovering cells by approximately 3- and 1.4-fold, respectively, when compared with the controls (*P*<0.01). Corresponding increased protein levels of ALKBH2 were observed (Figure 2B), but not in REV1 (data not shown). The kinetics of *ALKBH2* gene expression was further investigated by quantitative RT–PCR. The mRNA level was evidently induced from 0.5 h and remained high at 12 h (Figure 2C). The corresponding ALKBH2 protein was also elevated in a time-dependent manner (Figure 2D). Up-regulation of ALKBH2 at the protein level, but not at the RNA level, was found in DC group. Increase in ALKBH2 translation in DC group may be due to the small amount of DNA damage induced by the dark toxicity of Photofrin (see Figure 1).

### Knockdown of *ALKBH2* significantly increases the cytotoxicity of Ph-PDT

Compared with the control cells (transfected with Lipofectamine alone or negative control RNA), siALKBH2 cells had much reduced ALKBH2 protein expression (Figure 3A). The sensitivity of these cells to Photofrin was more than those of the control cells, resulting in more cell deaths after light irradiation (Figure 3B). The sensitising effect was more evident with increasing light doses, with a cytotoxicity at ∼8% at low light dose (0.8 J cm^−2^) and increased to ∼25% at high light dose (1.3 J cm^−2^). The cytotoxicity levels did not reach the respective LD 10 and LD 40 levels because the uptake of Photofrin was reduced in the presence of Lipofectamine (data not shown).

### Ph-PDT increases the expression of TP53 transcription factor and its activated phosphorylated form – p-TP53

To investigate the induction of *ALKBH2* gene expression under Ph-PDT condition, transcription factor-binding sites on *ALKBH2* were predicted and assessed. According to the Transcription Element Search System (TESS) web tool (http://www.cbil.upenn.edu/cgi-bin/tess/tess?RQ=WELCOME), TP53 is one of the potential-binding transcription factors. Its function in Ph-PDT was first examined by RT–PCR and western blotting. The mRNA and protein expression of TP53 in U87 glioma cells were shown to be increased 0.5 h after PDT (Figure 4A). The protein expression was maximal at 0.5 and 3.5 h. The level of p-TP53, which is associated with DNA repair mechanisms, was also shown to increase from 3.5 to 12.5 h in PDT-treated glioma cells.

### Increased TP53 binding on *ALKBH2* after Ph-PDT treatment

To show whether TP53 is involved directly, through binding as a transcription factor, in the transcription of *ALKBH2* induced by Ph-PDT, the ChIP assay was used. Figure 4B clearly shows that TP53 binds to *ALKBH2* gene, as there was a PCR product in the TP53-immunoprecipitated sample of Ph-PDT-treated cells. Two TP53-binding sites (approximately −190 bp and −14 bp; +1 is transcription start site) were predicted by TESS. Real-time PCR was used to determine the binding position of TP53 on *ALKBH2* promoter sequence. Figure 4C confirms TP53 binding to *ALKBH2* as well as indicating its binding location at −190 bp (4.5-fold increase), but not at the −14 bp region.

## Discussion

Numerous studies have shown that Ph-PDT induces significant DNA damage (Woods *et al*, 2004; Saczko *et al*, 2008). Different types of DNA damage may be seen, including double-strand breaks, single-strand breaks, DNA base oxidation and cross-links (Nowis *et al*, 2005). As DNA damage is not directly linked to the cell death caused by PDT, little research has been conducted to investigate the involvement of DNA repair in PDT. However, Penning *et al* (1994) showed that the inhibition of a DNA repair enzyme (poly(ADP-ribose)polymerase) activity and the formation of irreversible DNA damage were correlated to the killing effect of hematoporphyrin derivative PDT in a murine fibroblast cell line; note that Photofrin is purified form of hematoporphyrin derivative. They suggested that the involvement of DNA damage and repair in PDT is cell-type dependent. Another study by Gupta *et al* (2003) illustrated that enhanced DNA repair lowered the micronuclei frequencies and thus increased the relative resistance to PDT. The DNA repair capacity is determined not only by cell type, but also the oxygen concentration and subcellular localisation of Photofrin. As glioma treatment using Ph-PDT is under clinical trial, the detailed DNA repair mechanism involved should be studied, so that the efficacy of Ph-PDT can be enhanced by preventing DNA repair-induced resistance.

On the basis of the knowledge gained from the studies mentioned above, our preliminary focus was to examine the participation of DNA damage and repair in a glioma cell line after Ph-PDT. Our results were consistent with other reports in that the amount of DNA damage is positively associated with PDT light dosage (Woods *et al*, 2004). The DNA damage is increased in Ph-PDT treatment groups (LD 10 and LD 40) when the PDT light dose was increased (Figure 1). The DNA damage in treatment groups are significantly different from the glioma cells treated with light only (LCs) and with Photofrin only (DC). It is clear from the results presented here that light only will not cause significant DNA damage. In the DC, DNA was damaged to a lesser extent when compared with the PDT-treated groups. The DNA damage in the DC may be due to the low dose of light coming from ambient lighting that affected the cells during the course of the experiments. As Photofrin is not localised in the nucleus to cause DNA damage, the increase of DNA damage in PDT-treated groups may be explained by the impairment of the nuclear membrane after light irradiation (Moan *et al*, 1990; Saczko *et al*, 2007b). Consequently, sensitised reactive molecules, including photoproducts, can enter the nucleus and damage DNA (Evensen and Moan, 1982).

The DNA repair efficiency was less effective in the low light dose (LD 10) treatment group than that in the high light dose (LD 40) group. As the DNA repair capacity of the cells should be the same, the difference in the efficiency may be resulted from different DNA repair kinetics being activated by different light doses. Although DNA damage was also found in DCs, the damage was completely repaired after 24 h. This may be due to the small amounts of DNA damage present in the DC cells, but the participation of another DNA repair kinetics cannot be excluded. As our data indicate that DNA repair mechanisms are triggered in the relatively resistant U87 glioma cells after 48 h of recovery from Ph-PDT, we used real-time quantitative RT–PCR to determine which DNA repair gene(s) might be involved. The expression of the *ALKBH2* gene of DNA damage reversal and, to a much lesser extent, the *REV1* gene of translesion synthesis were found to be induced (Figure 2). The results indicate that both DNA damage reversal and translesion synthesis mechanisms may have important functions in glioma cells resistant to Ph-PDT. The *REV1* gene is involved in translesion synthesis, and allows damaged DNA to be tolerated by replicative bypass. When translesion synthesis is triggered, DNA replicates with mutations or errors and thus DNA damage-induced mutagenesis occurs (Prakash *et al*, 2005). As *ALKBH2* is more significantly expressed in the relatively resistant glioma cells, we focused on the molecular process leading to induction of *ALKBH2* expression during Ph-PDT and its contribution to PDT resistance.

The *ALKBH2* gene is not significantly expressed in normal brain cells, but high levels are found in liver tissue and sexual organs (Duncan *et al*, 2002; Lee *et al*, 2005). It is responsible for repairing 1-methyladenine (1meA), 3-methylcytosine (3meC) and 1,N^6^-ethenoadenine (*ε*A) on double-stranded DNA by oxidative demethylation (Lee *et al*, 2005; Ringvoll *et al*, 2008). Cetica *et al* (2009) showed that *ALKBH2* is highly expressed in gliomas and suggested that this aberrant expression has a part in tumour cell resistance to cancer treatments. We also found an up-regulation of *ALKBH2* in glioma cells from 30 min to 48 h post-treatment with Ph-PDT. This observation may imply that the photosensitised reactive products in Ph-PDT produce 1meA, 3meC and/or *ε*A on DNA. Most DNA damage studies of Ph-PDT target DNA damage caused by oxidation. Here, we suggest that the photosensitised reactive products may also cause DNA methylation and lipid peroxidation to produce methylated DNA damage and ethenoadenine DNA lesions, respectively. Prolonged high expression of *ALKBH2* also indicates that it may modulate the responsiveness to Ph-PDT. To confirm a specific function of *ALKBH2* in affecting Ph-PDT response, we used a gene-knockdown approach. As illustrated in Figure 3, cytotoxicity of Ph-PDT is enhanced after silencing the *ALKBH2* gene. This is the first report to show that the expression of *ALKBH2* in glioma cells correlates to Ph-PDT resistance and DNA damage reversal.

The transcription factors involved in the transcription of *ALKBH2* remain unknown. However, we have shown increased TP53 binding on the *ALKBH2* promoter region, and the levels of TP53 and p-TP53 were rapidly increased after Ph-PDT. Therefore, TP53 appears to be critical in the regulation of *ALKBH2* gene expression. There is some evidence that TP53 is involved in PDT, but its exact function in cellular responsiveness is controversial. Mikes *et al* (2009) reported that TP53-dependent apoptosis affects PDT efficacy. The investigators showed that adenocarcinoma colon cancer cells expressing wild-type TP53 have lower clonogenic efficiency than the TP53-deficient cells after Hypericin-mediated PDT. This may be due to a higher incidence of apoptosis caused by up-regulation of TP53 expression leading to the expression of pro-apoptotic proteins. However, TP53 may also confer PDT resistance to cells, possibly through DNA repair mechanisms, as cells allowed to recover for 24 h had similar clonogenic potential as the TP53-deficient cells. Using another photosensitiser, m-THPC, Heinzelmann-Schwarz *et al* (2003) showed that TP53 is required for apoptosis and interacts with the DNA repair gene Ataxia Telangiectasia Mutated to have a function in apoptosis as well as in responding to DNA damage induced by m-THPC-PDT. Our results are in agreement with these studies and clearly show that TP53 is involved in Ph-PDT. Up-regulation of p-TP53 at Ser-15 is indicative of DNA damage (Maya *et al*, 2001), thus, DNA repair has an important function in Ph-PDT resistance.

Some *in vitro* studies on human colon carcinoma, immortalised Li–Fraumeni syndrome and promyelocytic leukaemia found that the cell lines with mutant TP53 have lower sensitivity to Ph-PDT than those with wild-type TP53. This may be due to a decrease in TP53-dependent apoptosis after Ph-PDT (Tong *et al*, 2000). However, Evans *et al* (1997) found that Ph-PDT-induced apoptosis was higher in the lymphoblastic cell line with mutant TP53 than that with wild-type TP53, although the cytotoxic effect of Ph-PDT on both cell lines were not different. Another important finding by the same group was that the mutagenicity induced by Ph-PDT in the cell line with mutant TP53 was higher. Therefore, the relationship between TP53 and Ph-PDT responsiveness seems to be cell-type dependent. As different glioma cell lines may possess different TP53 status as well as other genetic differences, the effect of TP53 and *ALKBH2* on the efficacy of Ph-PDT should be compared with other cell lines. In our case, the U87 glioma cell line has wild-type TP53 and it may be involved in conferring resistance to these cells against Ph-PDT through the activation of *ALKBH2* DNA repair gene. Hence, our findings will further gain knowledge on how to improve the efficacy of Ph-PDT on gliomas by inhibiting the expression of *ALKBH2*. Further research is required to elucidate the function of TP53 and other regulators in controlling *ALKBH2* expression after Ph-PDT.

## Figures and Tables

**Figure 1:** The DNA damage and repair in U87 glioma cells after Photofrin-mediated PDT; DNA damage was detected by the alkaline comet assay and quantified as DNA percentage in tail. Cells were collected 3 h (black bars) and 24 h (white bars) after Ph-PDT. Cells treated with Photofrin (1 *μ*g ml^−1^) alone (DC) or Photofrin-mediated PDT at 0.8 and 1.3 J cm^−2^ light doses, that is lethal dose 10 and 40 (LD 10 and LD 40), were significantly damaged when compared with the untreated control (CNT) and cells exposed to 0.8 and 1.3 J cm^−2^ light doses only (LC1 and LC2). Twenty-four hours after treatment, the DNA damages in DC, LD 10 and LD 40 were significantly repaired. Data obtained from three independent experiments are expressed as mean+s.d. and analysed using paired *t*-test (^***^P<0.001).

**Figure 2:** Photofrin-mediated PDT induces DNA repair gene expression. (**A**) Quantitative real-time RT–PCR of DNA repair genes at 48 h after Photofrin-mediated PDT. *ALKBH2* and *REV1* were significantly expressed in LD10 and LD 40; DC is used as reference sample and CNT is used to examine the background expression levels of different DNA repair genes in U87 glioma cells. Data are expressed as mean+s.d. and analysed using one-way ANOVA with Tukey's multiple comparison post-test of three independent experiments (^**^P<0.01). (**B**) Increased ALKBH2 protein levels in glioma cells at 48 h after Ph-PDT. (**C**) Quantitative real-time RT–PCR showed significant *ALKBH2* gene expression at different time points after Photofrin-mediated PDT at LD 10. The mRNA level was significantly increased when compared with that of CNT and DC. Data are expressed as mean+s.d. and analysed using two-way ANOVA with Bonferroni's post-test of three independent experiments (^***^ represents the whole curve of LD 10 group is significant compared with both DC and CNT with *P*< 0.001 at 0.5, 3.5 and 12.5 h and *P*<0.01 at 6.5 and 9.5 h). (**D**) Protein expression of ALKBH2 at different time points after Photofrin-mediated PDT treatment at LD 10.

**Figure 3:** Effects on Photofrin-mediated PDT cytotoxicity of U87 glioma cells after knockdown of *ALKBH2* gene expression. (**A**) ALKBH2 protein expression in cells transfected with Lipofectamine alone or with the antisense oligonucleotide (siRNA) for *ALKBH2* gene knockdown or unrelated oligonucleotide as negative control (Neg CNT). (**B**) Survival rate (%) of cells treated with Lipofectamine alone (Lipofectamine) (dashed line with squares), siRNA (triangles) and Neg CNT (circles) was assessed using the trypan-blue assay. Cells were exposed to different light doses alone (left panel) or treated with Ph-PDT (right panel). Both protein expression and survival rate were examined 3 h after Ph-PDT. Data are expressed as mean±s.d. and analysed using one-way ANOVA with Tukey's multiple comparison post-test of three independent experiments (^***^P<0.001).

**Figure 4:** Function of TP53 in DNA repair after Photofrin-mediated PDT. (**A**) Expression of TP53 and p-TP53 at different time points after Ph-PDT. The TP53 mRNA and protein expression were increased at 0.5 and 3.5 h when compared with that of untreated control (CNT) and cells treated with Photofrin alone (DC). p-TP53 levels increased from 3.5 h and reached a maximum at 6.5 h. (**B**) Chromatin immunoprecipitations (ChIPs) were performed using anti-rabbit IgG or anti-p53 antibodies and then analysed by conventional PCR. Input control was DNA sample without any immunoprecipitation. (**C**) ChIP samples analysed and quantified by real-time PCR on two TP53-binding sites at approximately −190 bp and −14 bp from the transcription start site. Data are expressed as mean+s.d. and analysed by using paired *t*-test of three independent experiments (^***^P<0.001).

**Table 1:** The validated TaqMan gene expression assays

**Primers**	**Assay ID**	**Interrogated sequence**	**Exon boundary**	**Assay location**	**Amplicon length (bp)**
(1) ALKBH2	Hs00419572_m1	NM_001001655.1	2–3	478	86
(2) REV1	Hs00249411_m1	NM_001037872.1	2–3	268	63
(3) RAD52	Hs00172536_m1	NM_134424.2	2–3	197	65
(4) APEX1	Hs00172396_m1	NM_080648.1	3–4	510	81
(5) XRCC1	Hs00959834_m1	NM_006297.2	4–5	536	75
(6) ERCC5	Hs00164482_m1	NM_000123.2	14–15	3407	118

Adapted and modified from http://www.appliedbiosystems.com.hk/

**Table 2:** The primers used in conventional and real-time quantitative PCR for ChIP analysis

**Primers**	**Sequences (5′ to 3′)**	**Positions**	**Applications**
(1) p53_F1	TGCTCCCACTCGTGACAATA	−257 to −238	Used in conventional PCR and real-time PCR of position 1 p53-binding site.
(2) p53_R2	GCCACTGTCGAGAATCAC	−138 to −155	Used in real-time PCR of position 1 p53-binding site only.
(3) p53_F2	CAGCCGTGATTCTCGACA	−143 to −160	Used in real-time PCR of position 2 p53-binding site only.
(4) p53_R1	AACCGCACGCAAAATTCTGATAT	+147 to +125	Used in conventional PCR and real-time PCR of position 2 p53-binding site.

Abbreviations: ChIP=chromatin immunoprecipitation; PCR=polymerase chain reaction.

## References

[bib1] Adams K, Rainbow AJ, Wilson BC, Singh G (1999) *In vivo* resistance to photofrin-mediated photodynamic therapy in radiation-induced fibrosarcoma cells resistant to *in vitro* Photofrin-mediated photodynamic therapy. J Photochem Photobiol B 49: 136–1411039246310.1016/s1011-1344(99)00047-0

[bib2] Au CM, Luk SK, Jackson CJ, Ng HK, Yow CM, To SS (2006) Differential effects of photofrin, 5-aminolevulinic acid and calphostin C on glioma cells. J Photochem Photobiol B 85: 92–1011682911710.1016/j.jphotobiol.2006.06.002

[bib3] Biel M (2006) Advances in photodynamic therapy for the treatment of head and neck cancers. Lasers Surg Med 38: 349–3551678892310.1002/lsm.20368

[bib4] Cetica V, Genitori L, Giunti L, Sanzo M, Bernini G, Massimino M, Sardi I (2009) Pediatric brain tumors: mutations of two dioxygenases (hABH2 and hABH3) that directly repair alkylation damage. J Neurooncol 94: 195–2011929048110.1007/s11060-009-9837-0

[bib5] Christmann M, Tomicic MT, Roos WP, Kaina B (2003) Mechanisms of human DNA repair: an update. Toxicology 193: 3–341459976510.1016/s0300-483x(03)00287-7

[bib6] Collins AR, Dobson VL, Dusinska M, Kennedy G, Stetina R (1997) The comet assay: What can it really tell us? Mutat Res 375: 183–193920272810.1016/s0027-5107(97)00013-4

[bib7] Duncan T, Trewick SC, Koivisto P, Bates PA, Lindahl T, Sedgwick B (2002) Reversal of DNA alkylation damage by two human dioxygenases. Proc Natl Acad Sci USA 99: 16660–166651248623010.1073/pnas.262589799PMC139200

[bib8] Dysart JS, Patterson MS (2005) Characterization of Photofrin photobleaching for singlet oxygen dose estimation during photodynamic therapy of MLL cells *in vitro*. Phys Med Biol 50: 2597–26161590195710.1088/0031-9155/50/11/011

[bib9] Evans HH, Horng MF, Ricanati M, Deahl JT, Oleinick NL (1997) Mutagenicity of photodynamic therapy as compared to UVC and ionizing radiation in human and murine lymphoblast cell lines. Photochem Photobiol 66: 690–696938399210.1111/j.1751-1097.1997.tb03208.x

[bib10] Evensen JF, Moan J (1982) Photodynamic action and chromosomal damage: a comparison of haematoporphyrin derivative (HpD) and light with X-irradiation. Br J Cancer 45: 456–465707393910.1038/bjc.1982.74PMC2010917

[bib11] Ferrario A, Rucker N, Wong S, Luna M, Gomer CJ (2007) Survivin, a member of the inhibitor of apoptosis family, is induced by photodynamic therapy and is a target for improving treatment response. Cancer Res 67: 4989–49951751043010.1158/0008-5472.CAN-06-4785

[bib12] Frosina G (2009) DNA repair and resistance of gliomas to chemotherapy and radiotherapy. Mol Cancer Res 7: 989–9991960900210.1158/1541-7786.MCR-09-0030

[bib13] Fukushima T, Takeshima H, Kataoka H (2009) Anti-glioma therapy with temozolomide and status of the DNA-repair gene MGMT. Anticancer Res 29: 4845–485420032445

[bib14] Gerstner ER, Fine RL (2007) Increased permeability of the blood-brain barrier to chemotherapy in metastatic brain tumors: establishing a treatment paradigm. J Clin Oncol 25: 2306–23121753817710.1200/JCO.2006.10.0677

[bib15] Gupta S, Dwarakanath BS, Muralidhar K, Jain V (2003) Cellular uptake, localization and photodynamic effects of haematoporphyrin derivative in human glioma and squamous carcinoma cell lines. J Photochem Photobiol B 69: 107–1201263398310.1016/s1011-1344(02)00408-6

[bib16] Heinzelmann-Schwarz V, Fedier A, Hornung R, Walt H, Haller U, Fink D (2003) Role of p53 and ATM in photodynamic therapy-induced apoptosis. Lasers Surg Med 33: 182–1891294994810.1002/lsm.10213

[bib17] Hornung R, Walt H, Crompton NE, Keefe KA, Jentsch B, Perewusnyk G, Haller U, Kochli OR (1998) m-THPC-mediated photodynamic therapy (PDT) does not induce resistance to chemotherapy, radiotherapy or PDT on human breast cancer cells *in vitro*. Photochem Photobiol 68: 569–5749796440

[bib18] Jiang F, Robin AM, Katakowski M, Tong L, Espiritu M, Singh G, Chopp M (2003) Photodynamic therapy with photofrin in combination with buthionine sulfoximine (BSO) of human glioma in the nude rat. Lasers Med Sci 18: 128–1331450519510.1007/s10103-003-0269-3

[bib19] Lee DH, Jin SG, Cai S, Chen Y, Pfeifer GP, O’Connor TR (2005) Repair of methylation damage in DNA and RNA by mammalian AlkB homologues. J Biol Chem 280: 39448–394591617476910.1074/jbc.M509881200

[bib20] Livak KJ, Schmittgen TD (2001) Analysis of relative gene expression data using real-time quantitative PCR and the 2(-Delta Delta C(T)) method. Methods 25: 402–4081184660910.1006/meth.2001.1262

[bib21] Maya R, Balass M, Kim ST, Shkedy D, Leal JF, Shifman O, Moas M, Buschmann T, Ronai Z, Shiloh Y, Kastan MB, Katzir E, Oren M (2001) ATM-dependent phosphorylation of Mdm2 on serine 395: role in p53 activation by DNA damage. Genes Dev 15: 1067–10771133160310.1101/gad.886901PMC312683

[bib22] Mikes J, Koval J, Jendzelovsky R, Sackova V, Uhrinova I, Kello M, Kulikova L, Fedorocko P (2009) The role of p53 in the efficiency of photodynamic therapy with hypericin and subsequent long-term survival of colon cancer cells. Photochem Photobiol Sci 8: 1558–15671986241410.1039/b9pp00021f

[bib23] Moan J, Berg K, Kvam E (1990) Effects of photodynamic treatment on DNA and DNA-related cell functions. In Photodynamic Therapy of Neoplastic Disease Kessel D (ed), pp 197–209. CRC Press: Boston

[bib24] Nowis D, Makowski M, Stoklosa T, Legat M, Issat T, Golab J (2005) Direct tumor damage mechanisms of photodynamic therapy. Acta Biochim Pol 52: 339–35215990919

[bib25] Nyst HJ, Tan IB, Stewart FA, Balm AJ (2009) Is photodynamic therapy a good alternative to surgery and radiotherapy in the treatment of head and neck cancer? Photodiagnosis Photodyn Ther 6: 3–111944736610.1016/j.pdpdt.2009.03.002

[bib26] O’Connor AE, Gallagher WM, Byrne AT (2009) Porphyrin and nonporphyrin photosensitizers in oncology: preclinical and clinical advances in photodynamic therapy. Photochem Photobiol 85: 1053–10741968232210.1111/j.1751-1097.2009.00585.x

[bib27] Penning LC, Lagerberg JW, VanDierendonck JH, Cornelisse CJ, Dubbelman TM, VanSteveninck J (1994) The role of DNA damage and inhibition of poly(ADP-ribosyl)ation in loss of clonogenicity of murine L929 fibroblasts, caused by photodynamically induced oxidative stress. Cancer Res 54: 5561–55677923197

[bib28] Pervaiz S (2001) Reactive oxygen-dependent production of novel photochemotherapeutic agents. FASEB J 15: 612–6171125937910.1096/fj.00-0555rev

[bib29] Prakash S, Johnson RE, Prakash L (2005) Eukaryotic translesion synthesis DNA polymerases: specificity of structure and function. Annu Rev Biochem 74: 317–3531595289010.1146/annurev.biochem.74.082803.133250

[bib30] Rigual NR, Thankappan K, Cooper M, Sullivan MA, Dougherty T, Popat SR, Loree TR, Biel MA, Henderson B (2009) Photodynamic therapy for head and neck dysplasia and cancer. Arch Otolaryngol Head Neck Surg 135: 784–7881968739910.1001/archoto.2009.98PMC2810853

[bib31] Ringvoll J, Moen MN, Nordstrand LM, Meira LB, Pang B, Bekkelund A, Dedon PC, Bjelland S, Samson LD, Falnes PO, Klungland A (2008) AlkB homologue 2-mediated repair of ethenoadenine lesions in mammalian DNA. Cancer Res 68: 4142–41491851967310.1158/0008-5472.CAN-08-0796PMC4725713

[bib32] Saczko J, Chwilkowska A, Kulbacka J, Berdowska I, Zielinski B, Drag-Zalesinska M, Wysocka T, Lugowski M, Banas T (2008) Photooxidative action in cancer and normal cells induced by the use of photofrin in photodynamic therapy. Folia Biol (Praha) 54: 24–291822636210.14712/fb2008054010024

[bib33] Saczko J, Kulbacka J, Chwilkowsa A, Pola A, Lugowski M, Marcinkowska A, Malarska A, Banas T (2007a) Cytosolic superoxide dismutase activity after photodynamic therapy, intracellular distribution of Photofrin II and hypericin, and P-glycoprotein localization in human colon adenocarcinoma. Folia Histochem Cytobiol 45: 93–9817597022

[bib34] Saczko J, Mazurkiewicz M, Chwilkowska A, Kulbacka J, Kramer G, Lugowski M, Snietura M, Banas T (2007b) Intracellular distribution of Photofrin in malignant and normal endothelial cell lines. Folia Biol (Praha) 53: 7–121732883710.14712/fb2007053010007

[bib35] Stylli SS, Howes M, MacGregor L, Rajendra P, Kaye AH (2004) Photodynamic therapy of brain tumours: evaluation of porphyrin uptake versus clinical outcome. J Clin Neurosci 11: 584–5961526122610.1016/j.jocn.2004.02.001

[bib36] Szabo SE, Monroe SL, Fiorino S, Bitzan J, Loper K (2004) Evaluation of an automated instrument for viability and concentration measurements of cryopreserved hematopoietic cells. Lab Hematol 10: 109–11115224767

[bib37] Tong Z, Singh G, Rainbow AJ (2000) The role of the p53 tumor suppressor in the response of human cells to photofrin-mediated photodynamic therapy. Photochem Photobiol 71: 201–2101068739510.1562/0031-8655(2000)071<0201:trotpt>2.0.co;2

[bib38] Usuda J, Hirata T, Ichinose S, Ishizumi T, Inoue T, Ohtani K, Maehara S, Yamada M, Tsutsui H, Okunaka T, Kato H, Ikeda N (2008) Tailor-made approach to photodynamic therapy in the treatment of cancer based on Bcl-2 photodamage. Int J Oncol 33: 689–69618813781

[bib39] Usuda J, Tsunoda Y, Ichinose S, Ishizumi T, Ohtani K, Maehara S, Ono S, Tsutsui H, Ohira T, Okunaka T, Furukawa K, Sugimoto Y, Kato H, Ikeda N (2010) Breast cancer resistant protein (BCRP) is a molecular determinant of the outcome of photodynamic therapy (PDT) for centrally located early lung cancer. Lung Cancer 67: 198–2041947703210.1016/j.lungcan.2009.04.002

[bib40] Woods JA, Traynor NJ, Brancaleon L, Moseley H (2004) The effect of photofrin on DNA strand breaks and base oxidation in HaCaT keratinocytes: a comet assay study. Photochem Photobiol 79: 105–11314974722

[bib41] Zheng X, Jiang F, Katakowski M, Zhang X, Jiang H, Zhang ZG, Chopp M (2008) Sensitization of cerebral tissue in nude mice with photodynamic therapy induces ADAM17/TACE and promotes glioma cell invasion. Cancer Lett 265: 177–1871835860010.1016/j.canlet.2008.02.023PMC2432085

